# Plasma Resolvin D2 to Leukotriene B_4_ Ratio Is Reduced in Diabetic Patients with Ischemic Stroke and Related to Prognosis

**DOI:** 10.1155/2021/6657646

**Published:** 2021-02-26

**Authors:** Zhijuan Miao, Xin Tang, Marianne Schultzberg, Yuwu Zhao, Xiuzhe Wang

**Affiliations:** ^1^Department of Neurology, Shanghai Jiao Tong University Affiliated Sixth People's Hospital, Shanghai, China; ^2^Department of Neurobiology, Care Sciences and Society, Center for Alzheimer Research, Karolinska Institutet, Stockholm, Sweden

## Abstract

**Background:**

Diabetes mellitus (DM) aggravates symptoms and prognosis of acute ischemic stroke (AIS), and inflammation plays an important role therein. Resolvin D2 (RvD2) is one of the specialized pro-resolving mediators (SPMs), while leukotriene B_4_ (LTB_4_) is a classic proinflammatory mediator. The ratio of RvD2 to LTB_4_ is an index of pro-resolving/proinflammatory balance. We aim to explore the role of RvD2/LTB_4_ ratio in ischemic stroke complicated with DM.

**Methods:**

The plasma levels of RvD2 and LTB_4_ were analyzed by enzyme immunoassay in stroke patients with DM (DM + AIS group) or without DM (nonDM+AIS group). Patients were followed up at 90 days after stroke onset, and modified Rankin Score (mRS) was assessed. The association of RvD2/LTB_4_ ratio with stroke severity and prognosis was also analyzed.

**Results:**

The plasma levels of RvD2 were positively correlated to LTB_4_. The RvD2/LTB_4_ ratio in DM + AIS group was lower than that in the nonDM+AIS group. No correlation was found between the RvD2/LTB_4_ ratio and infarct size or NIHSS score. The RvD2/LTB_4_ ratio at baseline was significantly lower in the poor prognosis group (mRS ≥ 3) than that in the good prognosis group (mRS ≤ 2).

**Conclusions:**

Our study indicated that the balance between pro-resolving and proinflammatory mediators was impaired by diabetes in ischemic stroke. The RvD2/LTB_4_ ratio may serve as a biomarker of prognosis for ischemic stroke.

## 1. Introduction

Diabetes mellitus (DM) is an independent risk factor for ischemic stroke and can treble the risk of cardiovascular and cerebrovascular diseases [1]. Inflammation plays an important role in the pathogenesis of diabetes. Pickup showed that cytokines mediate inflammatory response in type 2 diabetes and are directly involved in the development of DM and its vascular complications [2]. The use of salicylic acid or interleukin (IL-) 1 receptor antagonists in DM patients can lower blood glucose levels, further supporting the hypothesis that DM is an inflammatory disease [3]. Inflammation also plays a key role in the pathophysiology of ischemic stroke complicated with DM [4]. For example, matrix metalloproteinase-2 (MMP-2) activity, cyclooxygenase-2 (COX-2), IL-1*β*, and IL-6 were increased in the diabetic mouse brain after stroke [5–7].

Resolution of inflammation is the key program that regulates inflammation and ensures proinflammatory responses are not overactive. Uncontrolled inflammatory response and impaired resolution contribute to the pathological process of many diseases. In the past decade, specialized pro-resolving mediators (SPMs) have been identified as the central controllers of inflammation resolution. These small lipid molecules, including, e.g., lipoxins (LXs), resolvins (Rvs), protectins (PDs), and maresins (MaRs), monitor inflammation of resolution in a receptor-dependent manner [8]. The balance between proinflammatory mediators and SPMs regulates the duration of inflammatory response and the time course of homeostasis recovery. Imbalance between these two forces leads to the occurrence of inflammatory diseases. Leukotriene B_4_ (LTB_4_) is a classical proinflammatory lipid mediator derived from arachidonic acid (AA). The ratio of SPMs to LTB_4_ reflects the degree of the resolving-proinflammatory balance and has been studied in a variety of disease models. For example, it has been reported that the LXA_4_/LTB_4_ ratio decreased in alveolar lavage fluid of patients with cystic fibrosis, suggesting that disturbed resolution of inflammation contributes to the pathological changes of cystic fibrosis in the airway [9]. The ratio of RvD1/LTB_4_ and MaR1/LTB_4_ was reduced in preeclampsia compared to normal pregnancy, indicating that insufficient production of SPMs may be involved in the occurrence of preeclampsia [10]. Resolvin D2 (RvD2) is derived from docosahexaenoic acid (DHA). It has been shown that RvD2 can reduce infarct volume and dampen inflammation in experimental models of stroke [11, 12].

The RvD2/LTB_4_ ratio has been used as a biomarker for carotid intima thickness and plaque stability in cardiovascular disease [13, 14].

The aim of this study is to characterize the changes of RvD2/LTB_4_ ratio in DM patients with acute ischemic stroke. We also explored possible associations between the RvD2/LTB_4_ ratio and clinical characteristics of the patients, as well as the relationship of RvD2/LTB_4_ ratio and stroke prognosis.

## 2. Methods

### 2.1. Study Population and Clinical Data Collection

We enrolled 57 patients with acute ischemic stroke from the Department of Neurology, Shanghai Jiao Tong University Affiliated Sixth People's Hospital. According to the combination of DM, the patients were divided into two groups: non-DM patients with acute ischemic stroke (nonDM+AIS group) and DM patients with acute ischemic stroke (DM + AIS group). Patients with coma, severe cardiac/hepatic/renal dysfunction, mental illness, history of other endocrine diseases, tumor, or autoimmune disease were excluded from the study. Patients who had acute systematic inflammatory disease within 1 month or received fibrinolytic thrombolysis were also excluded. All stroke patients met the diagnostic criteria of Chinese guidelines for the diagnosis and treatment of acute ischemic stroke 2014 [15] and were confirmed by computed tomography (CT) or magnetic resonance imaging (MRI). All DM patients met the diagnostic criteria made by the European Diabetes Policy Group for type 2 diabetes [16]. The patients were followed up at 90 days after stroke onset, and the modified Rankin Score (mRS) was assessed.

General information was collected covering age, gender, smoking/drinking history, and medical history. Routine laboratory analyses including glycated hemoglobin (HbA1c), fasting blood glucose, triglyceride, cholesterol, high-density lipoprotein (HDL), low-density lipoprotein (LDL), serum uric acid, white blood cell count, and neutrophil count were performed following routine procedures in the Department of Laboratory Medicine of Shanghai Jiao Tong University Affiliated Sixth People's Hospital. All participants or their authorized caregivers signed an informed consent. The study was approved by the ethical committee of Shanghai Jiao Tong University Affiliated Sixth People's Hospital.

### 2.2. Blood Sampling and Enzyme Immunoassay Analysis

Fasting blood samples were collected in EDTA anticoagulant tubes by venipuncture from all participants. All samples were taken within 72 h after disease onset. The samples were then centrifuged immediately, and the resulting plasma was stored at -80°C until further processing. Endogenous concentrations of RvD2 and LTB_4_ in plasma were determined by enzyme immunoassay (EIA) kits (Cayman Chemical, MI, USA). The collected plasma samples underwent a purification procedure according to the instructions of the EIA kits. Briefly, C18 Sep-Pak® light columns (Waters Corporation, MA, USA) were conditioned by methanol and water. The plasma samples were acidified to pH 4.0 (for LTB_4_) or pH 5.0 (for RvD2) and injected into the preconditioned C18 column. Subsequently, the columns were washed with distilled water, and the purified samples were eluted with 1% methanol in ethyl acetate (for LTB_4_) or methanol (for RvD2). The samples were then dried by N_2_ gas and resuspended in EIA buffer for assessment of RvD2 and LTB_4_ according to the specific instructions for the kits.

### 2.3. Statistical Analysis

All statistical analyses were performed using the IBM SPSS software (version 22, SPSS Inc., USA). Continuous and parametric variables were expressed as mean ± standard deviation (SD), and nonparametric distributed variables were expressed as median (IQR) and 25th-75th percentiles. Categorical variables were expressed as percentages. Differences between the two groups were compared by Mann–Whitney *U* test for nonparametric variables, and *χ*^2^ or Fisher's exact test was used for categorical variables. Spearman correlation analysis was performed to evaluate the possible associations of lipid mediator with clinical or laboratory parameters. Receiver operating characteristic (ROC) curves and area under the curves (AUC) were calculated to evaluate the predictive power of the RvD2/LTB_4_ ratio for stroke outcome. *p* < 0.05 was considered as significant in all statistical analyses.

## 3. Results

### 3.1. Clinical Characteristics

A total of 57 cases were enrolled, including 25 nondiabetic patients with acute ischemic stroke (nonDM+AIS group) and 32 diabetic patients with acute ischemic stroke (DM + AIS group). There was no significant difference in age, history of smoking, drinking, hypertension, and atrial fibrillation between the two groups. The levels of HbA1c and fasting blood glucose were higher in the diabetic group than in the nondiabetic group (Table 1). There was no significant difference with regard to other laboratory tests, including triglycerides, cholesterol, HDL, LDL, serum uric acid, white blood cell count, and neutrophil count.

### 3.2. Plasma Levels of RvD2, LTB_4_, and Their Ratio in DM + AIS and nonDM+AIS Groups

There was no significant difference between the two groups with regard to plasma RvD2 concentration (Figure 1(a)). LTB_4_ levels in the DM + AIS group were higher than that in the nonDM+AIS group (Figure 1(b)). To evaluate the balance of pro-resolving lipid mediators and pro-inflammation lipid mediators, we calculated the RvD2/LTB_4_ ratio. The DM + AIS group had a lower RvD2/LTB_4_ ratio than the nonDM+AIS group (Figure 1(c)). A positive correlation was found between RvD2 and LTB_4_ levels (*r* = 0.262, *p* = 0.049) (Figure 1(d)).

### 3.3. Association of Infarct Volume/NIHSS Score with RvD2/LTB_4_ Ratio

Diffusion-weighted MRI was used to assess infarct volume. The volume of cerebral infarction was calculated according to the Pullicino formula (length × width × layer/2, cm^3^) [17]. The stroke patients were divided into small infarct (<5 cm^3^, *n* = 29), medium infarct (5-10 cm^3^, *n* = 7), and large infarct (>10 cm^3^, *n* = 19). There was no significant difference in RvD2/LTB_4_ ratio between the three groups (Figure 2(a)). The NIHSS score was used to evaluate the degree of neurological impairment on the first day of admission. The patients were divided into three groups, including mild neurological impairment (NIHSS score < 4, *n* = 28), moderate neurological impairment (NIHSS score 4-15, *n* = 25), and severe neurological impairment (NIHSS score > 15, *n* = 4). We found that there was a gradient trend of decrease of RVD2/LTB_4_ ratio from mild to severe neurological impairment, though not statistically significant (Figure 2(b)).

### 3.4. Relationship between the Ratio of RvD2/LTB_4_ and Stroke Prognosis

According to the 90-day mRS score, the patients were divided into the good prognosis group (mRS ≤ 2, *n* = 36) and poor prognosis group (mRS ≥ 3, *n* = 21). We found that baseline RvD2/LTB_4_ ratio in the good prognosis group was higher than that in the poor prognosis (0.85[0.42–1.17] vs. 0.58 [0.28–0.77], *p* = 0.040) (Figure 2(c)). Correlation analysis showed that the RvD2/LTB_4_ ratio was negatively correlated with the mRS score (Spearman's rho test, *r* = −0.291, *p* = 0.028) (Figure 2(d)). ROC curve analysis revealed that RvD2/LTB_4_ produced an unsatisfactory area under the curve (AUC = 0.664) for predicting stroke prognosis with a 95% confidence interval of 0.527–0.784, *p* = 0.025. The associated criterion was 0.63 with 76.2% specificity and 58.3% sensitivity (Figure 3).

## 4. Discussion

In the present study, the RvD2/LTB_4_ ratio was significantly reduced in DM stroke patients compared to non-DM stroke diabetic patients, indicating that DM impairs the balance between pro-resolving and proinflammatory signals in ischemic stroke. Furthermore, the RvD2/LTB_4_ ratio in the acute stage of ischemic stroke was correlated with patient prognosis. These results provided novel potential mechanisms in excessive inflammation in DM patients with ischemic stroke.

Inflammation is a key program that mediates pathogenic and pathological effects of DM on ischemic stroke [4, 18]. The levels of circulating proinflammatory cytokines, such as tumor necrosis factor-*α* (TNF-*α*) and IL-1, are increased in DM patients [19]. Sitagliptin was applied in the treatment of diabetes mellitus type 2. Studies have shown that sitagliptin has a neuroprotective effect by reducing neuroinflammation [20]. Atorvastatin could decrease the concentration of IL-6 and TNF-*α* and improved the outcome of ventilator-associated pneumonia in patients with ischemic stroke [21]. Herrera et al. demonstrated that RvE1 increased the neutrophil phagocytosis of *P. gingivalis* in WT animals but had no impact in diabetes animals. In RvE1 receptor-transgenic diabetic mice, the impaired neutrophil phagocytosis ability was rescued by RvE1 [22]. Above all, the proresolution system appears to be compromised in DM. This may explain why diabetic patients with ischemic stroke have more severe symptoms and prognosis. Parlapiano et al. demonstrated that diabetic patients have increased levels of LTB_4_ and activity of polymorphonuclear leukocyte, and this activation is correlated to glycated hemoglobin level [23].

Overactivated inflammation has been reported in the etiology of exaggerated brain damage in diabetic stroke models [24, 25]. Effective resolution of inflammation is essential for balancing poststroke inflammation to restore homeostasis of the brain. SPMs promote the resolution of inflammation and the recovery of tissue homeostasis [8]. RvD2 has been shown to exert anti-inflammatory and pro-resolving properties in various disease models [12, 26, 27]. The levels of endogenous RvD2 were inconsistent in different disease models and at different stages of the disease. Zuo et al. reported that the experimental stroke led to a decrease of RvD2 in the brain [12]. In epilepsy, the levels of brain RvD2 were reduced after seizure [28]. Conversely, in a mouse model of acute lung injury, the levels of RvD2 were increased within 24 h of LPS-induced lung inflammation [29]. In a murine model of hind limb ischemia, RvD2 and 17-HDHA were generated robustly in the bone marrow as early as 24 h postsurgery [27]. Thus, it is valuable to evaluate the balance of pro-resolving and proinflammatory signals in a comprehensive way. LTB_4_ is a classic inflammatory lipid mediator and has been implicated in ischemic stroke pathology [30, 31]. The levels of LTB_4_ in plasma increased rapidly after stroke in humans [30]. Early and sustained increase of LTB_4_ is associated with poor functional recovery of stroke [30]. High LTB_4_ levels were also associated with larger nonhealing lesion areas and increased bacterial load in skin wound of diabetic mice [32]. The ratio of SPMs/LTB_4_ has been considered as an index of the balance between pro-resolving and proinflammatory signals. For example, the ratios of plasma RvD1/LTB_4_ and MaR1/LTB_4_ were associated with inflammation status in preeclampsia [10]. In atherosclerosis, reduced salivary RvD1/LTB_4_ ratio was found to reflect an imbalance of pro-resolving and proinflammatory forces and could predict thicker carotid intima [13]. Moreover, an abnormal ratio of SPM/LTB_4_ was observed in the instable plaques derived from atherosclerosis patients [14].

In the present study, we utilized the plasma RvD2/LTB_4_ ratio as a possible indicator for poststroke inflammation. We found lower RvD2/LTB_4_ ratio in DM patients compared to non-DM patients. With ischemic stroke compared to nondiabetic patients. This may indicate that DM impairs the resolution of inflammation in acute ischemic stroke. Such an effect of DM in the resolution of inflammation has been shown in other diseases. For example, an imbalance of proinflammatory and pro-resolving mediators was observed in DM patients with tuberculosis [33]. A study on DM-associated retina damage showed that hyperglycemia may decrease RvD1 in the retina [34]. Furthermore, DM has been shown to impair the biosynthesis of PD1 and thus result in the overactivation of macrophages in wound healing [35]. These studies supported our finding that DM may disturb the resolution of inflammation in ischemic stroke.

We also explored the association of RvD2/LTB_4_ ratio with stroke severity and prognosis. We found no correlation between the RvD2/LTB_4_ ratio and infarct volume nor NIHSS score. This finding is consistent with previous publications showing that inflammation is not linearly associated with the degree of brain damage in stroke [31, 36, 37].

On the other hand, it has been shown that neuroendocrine biomarkers, such as copeptin and cortisol, are correlated with short-term outcome and mortality of ischemic stroke [38]. We found an association between plasma RvD2/LTB_4_ ratio and 90-day prognosis. Patients with poor prognosis had lower levels of RvD2/LTB_4_ ratio at baseline. The levels of pro-resolving activities at the acute phase may represent an overall capacity of the body to restore homeostasis after stroke. This is consistent with the previous report that high levels of circulating TNF-*α*, IL-6, and MMP-9 were associated with a poor prognosis in acute ischemic stroke [39–41]. The ROC curve analysis of the RvD2/LTB_4_ ratio for prognosis revealed an AUC of 0.664. Although the RvD2/LTB_4_ ratio may serve as a biomarker of stroke prognosis, the predictive power, specificity, and sensitivity are relatively low.

In summary, our data indicate that DM may disturb the balance between pro-resolving and proinflammatory mediators in ischemic stroke. Moreover, the reduced RvD2/LTB_4_ ratio in the acute phase of stroke may predict a poor prognosis. These findings provide new insights into the failure of resolution of inflammation in DM patients with ischemic stroke. Limitation of this study includes the small sample size, single center design, and no validation cohort. Larger sample sizes of patients from multiple centers are needed to validate our findings in future studies. In addition, studies involving animal and cellular models are essential to further elucidate the intrinsic mechanisms of resolution failure in DM patients with acute ischemic stroke.

## Figures and Tables

**Figure 1:** Plasma levels of RvD2, LTB_4_, and RvD2/LTB_4_ ratio in acute ischemic stroke. (a) Comparison of the plasma concentrations of RvD2 shows no difference in the nonDM+AIS group and DM + AIS group. (b) Plasma concentrations of LTB_4_ were increased in the nonDM+AIS group and nonDM+AIS group. (c) The RvD2/LTB_4_ ratio of the DM + AIS group was lower compared to that in the nonDM+AIS group. (d) Correlation analysis shows a positive association between RvD2 and LTB_4_ (Spearman rho test, *r* = 0.262, *p* = 0.049). Error bars represent IQR. ns: none significant. ^∗^*p* < 0.05. DM: diabetes mellitus; AIS: acute ischemic stroke; LTB_4_: leukotriene B_4_; RvD2: resolvin D2.

**Figure 2:** The association of RvD2/LTB_4_ ratio with infarct volume, NIHSS score, and 90-day prognosis. (a) Ratios of plasma RvD2/LTB_4_ were not different in the small, medium, and large infarct volume group. (b) Ratios of plasma RvD2/LTB_4_ were not different in mild, moderate, and severe neurological deficit groups. (c) Ratios of plasma RvD2/LTB_4_ in good prognosis were higher compared with that in the poor prognosis group. (d) There was a negative association of RvD2/LTB_4_ ratio with 90-day mRS (Spearman rho test, *r* = −0.291, *p* = 0.028). Error bars represent IQR. ns: none significant. ^∗^*p* < 0.05. LTB_4_: leukotriene B_4_; mRS: modified Rankin Scale; NIHSS: National Institutes of Health Stroke Scale; RvD2: resolvin D2.

**Figure 3:** Possible predictive role of RvD2/LTB_4_ in stroke prognosis. ROC curve analysis showed AUC = 0.664 with a 95% confidence interval of 0.527–0.784, *p* = 0.025. The associated criterion was 0.63 with 76.2% specificity and 58.3% sensitivity. AUC: area under the curve; LTB_4_: leukotriene B_4_; ROC: receiver operating characteristic curves; RvD2: resolvin D2.

**Table 1:** Baseline characteristics of the patients.

	nonDM+AIS (*n* = 25)	DM + AIS (*n* = 32)	*p*
Age	66.36 ± 9.50	69.31 ± 9.89	0.260
Gender (male)	19 (76)	24 (75)	0.931
Smoking	8 (32)	6 (18.8)	0.249
Alcohol use	4 (16)	4 (12.5)	0.706
Hypertension	17 (68)	26 (81.3)	0.249
Atrial fibrillation	3 (12)	5 (15.6)	0.995
HbA1c	5.80 (5.50-6.05)	7.55 (6.90-9.23)	<0.01
Fasting blood glucose/mmol/L	5.31 (4.88-6.31)	7.82 (6.67-9.58)	<0.01
Triglyceride/mmol/L	4.63 (3.48-5.58)	4.50 (3.44-5.75)	0.803
Cholesterol/mmol/L	1.63 (1.21-2.17)	1.59 (1.02-3.08)	0.923
HDL/mmol/L	1.13 (0.81-1.31)	0.98 (0.87-1.20)	0.705
LDL/mmol/L	3.08 ± 1.01	3.09 ± 0.86	0.975
Uric acid/umol/L	346 (326-361)	321 (259-354)	0.061
White blood cell count × 10^9^/L	7.20 (5.75-9.05)	6.95 (5.95-8.68)	0.994
Neutrophils cell count × 10^9^/L	4.20 (3.10-5.90)	4.90 (3.83-6.88)	0.228

Data are presented as mean ± SD or median ± IQR or *n* (%). DM: diabetes mellitus group; HDL: high-density lipoprotein; AIS: acute ischemic stroke; LDL: low-density lipoprotein.

## Data Availability

The data used to support the findings of this study are available from the corresponding authors upon request.
